The article "Efficacy and Prognosis of Ultrasound-Guided Percutaneous Catheter Drainage in Patients with Liver Abscess Complicated with Septic Shock" was retracted in 2023. Reasons: signs of a paper mill; suspected computer-generated content; unreliable results or conclusions; lack of ethics approval or compliance.

# Efficacy and Prognosis of Ultrasound-Guided Percutaneous Catheter Drainage in Patients with Liver Abscess Complicated with Septic Shock

**DOI:** 10.1155/2022/4688356

**Published:** 2022-07-06

**Authors:** Shoulin Li, Jiye Luo, Zheng Wang, Chunyang Lv, Yang Wang

**Affiliations:** ^1^Department of Emergency Medicine, The First People's Hospital of Lianyungang (The First Affiliated Hospital of Kangda College of Nanjing Medical University), Lianyungang City, Jiangsu Province 222061, China; ^2^Department of Hepatobiliary Surgery, Huai'an Second People's Hospital (The Affiliated Huai'an Hospital of Xuzhou Medical University), Huai'an, Jiangsu 223000, China

## Abstract

**Objective:**

Currently, the therapeutic effect and outcomes of US-PCD in patients with liver abscess and septic shock remain unclear. This study is aimed at investigating the effects of ultrasound-guided percutaneous catheter drainage (US-PCD) on the prognosis of patients with liver abscess complicated with septic shock.

**Method:**

We retrieved and assessed the data of 120 patients with liver abscess complicated with septic shock diagnosed at our hospital from January 2019 to March 2021. The patients underwent US-PCD in the observation group or conventional surgical incision and drainage in the control group. After treatment, we determined the levels of liver function indicators alanine aminotransferase (ALT), aspartate aminotransferase (AST), total bilirubin (TBIL), direct bilirubin (DBIL), and alkaline phosphatase (ALP) as well as the levels of inflammatory cytokines IL-6, IL-8, and TNF-*α* in serum using ELISA on postoperative days 0, 2, 4, and 6. The postoperative body temperature recovery, peripheral white blood cell count recovery, extubation, postoperative length of stay, and complications were recorded, with a 12-month follow-up to calculate their survival rate.

**Results:**

After treatment, the ALT, AST, TBIL, DBIL, and ALP levels and inflammatory factor levels in the two groups were gradually reduced over time and returned to the normal range with a better recovery trend in the observation group. US-PCD was associated with better postoperative body temperature recovery, peripheral white blood cell count recovery, shorter extubation time, hospital stay, lower postoperative rate, and a higher survival rate.

**Conclusion:**

US-PCD may be effective in treating liver abscess and can significantly improve the prognosis of patients.

## 1. Introduction

A liver abscess is defined as a mass filled with pus in the liver due to an injury or intra-abdominal infection disseminated from the portal circulation [1]. It may occur due to infections and from the bloodstream as the liver receives blood from both the system and portal circulations [2]. Common pathophysiology for developing liver abscesses could be leakage of bowel contents, peritonitis, appendicitis, and cholangitis [3, 4]. Various microorganisms can cause suppurative liver lesions and can be divided into bacterial liver abscess, fungal liver abscess, and amoebic liver abscess. Bacterial liver abscess is the most frequently encountered, with *Escherichia coli* and *Staphylococcus aureus* being its main pathogenic bacteria. If not treated in time, this disorder can cause systemic toxic infections, leading to death, with a mortality rate of up to 10%–30% [5, 6]. Due to its nonspecific clinical characteristics, a liver abscess is usually not effectively diagnosed at an early stage. Missing opportunities for early diagnosis and treatment triggers the rapid progression of septic shock [7], leading to organ failure and, ultimately, death. Studies have shown that 16% of patients with liver abscesses suffer from septic shock, and death occurs in 2.2% of them [8]. Presently, the preferred liver abscess treatments include percutaneous transhepatic puncture and drainage and broad-spectrum antibiotics [9]. However, broad-spectrum antibiotics may lead to drug resistance in patients [10].

The article "Efficacy and Prognosis of Ultrasound-Guided Percutaneous Catheter Drainage in Patients with Liver Abscess Complicated with Septic Shock" was retracted in 2023. Reasons: signs of a paper mill; suspected computer-generated content; unreliable results or conclusions; lack of ethics approval or compliance.

In recent years, with great advances in imaging techniques, such as interventional ultrasound technology, the diagnosis and treatment of liver abscess has undergone fundamental changes. Percutaneous transhepatic abscess aspiration and drainage have gradually replaced the traditional surgical drainage [11, 12]. This novel treatment has the advantages of less trauma, short course of treatment, and low cost, especially suitable for patients with diabetes and frail and elder patients, and can further reduce the risks of complications and mortality in these patients [13]. Ultrasound (US) is considered a reliable guidance system for percutaneous catheter drainage (PCD) [14] and has been used to treat abscesses at various body locations such as the pancreas, retroperitoneum, and spleen [15–18]. However, the therapeutic effect and prognosis of US-PCD on liver abscesses with septic shock are still unclear. Therefore, in this study, we used different treatments for patients with liver abscesses to investigate the therapeutic effect of US-PCD and to provide a research direction for the effective treatment of liver abscesses in clinical practice.

## 2. Materials and Methods

### 2.1. Clinical Data

The data of 120 patients with liver abscess complicated with septic shock diagnosed at our hospital from January 2019 to March 2021 were retrieved and analyzed. They were classified into an observation group (*n* = 70) and a control group (*n* = 50) based on whether they received US-PCD or routine surgical incision and drainage, respectively. The study inclusion criteria were as follows: (1) patients were diagnosed with liver abscess by enhanced computed tomography (CT) or magnetic resonance imaging before operation and were confirmed as liver abscess by liver puncture or surgery; (2) patients with normal coagulation function; (3) preoperative complete blood routine, liver, and kidney function, related tumor markers, electrocardiogram, chest X-ray, and other examinations; (4) no serious heart, lung, liver, kidney, and other important organ diseases; (5) patients with no communication disorders and no abnormal mental behavior; (6) in case of no typical imaging and etiological evidence, patients had abscess shrinking or disappearing, and their symptoms were improved after antibiotic treatment. The exclusion criteria were as follows: (1) amebic liver abscess, tuberculous liver abscess, and other liver inflammatory diseases; (2) ruptured abscess resulting in peritonitis, subphrenic abscess, or empyema; (3) cirrhosis, malignant tumors, and massive ascites; (4) interventional treatment was converted to surgery after failure; and (5) poor coagulation function, mental illness, severe cognitive impairment, or language problems. The general data of the included patients were recorded. All patients signed the informed consent form for surgical treatment, and this study was approved by the Ethics Committee of Huai'an Second People's Hospital (HEYLL201856).

The article "Efficacy and Prognosis of Ultrasound-Guided Percutaneous Catheter Drainage in Patients with Liver Abscess Complicated with Septic Shock" was retracted in 2023. Reasons: signs of a paper mill; suspected computer-generated content; unreliable results or conclusions; lack of ethics approval or compliance.

### 2.2. Treatment Methods

The observation group was treated with US-PCD. Color Doppler ultrasound diagnostic apparatus was used for the patients, and the needle insertion path was determined by first placing the patients in a left lateral decubitus position. After identification of the insertion path, disinfection and draping were performed, and 3% lidocaine was applied to complete local anesthesia. A 3 mm incision was made in the skin with a blade, and the puncture was completed under ultrasound guidance. An 8-11 F percutaneous transhepatic biliary drainage tube was inserted into the abscess cavity with a pigtail drainage tube, the needle core pulled out, the drainage bag connected, and the wound bandaged. After surgery, US was repeated every 3 days until the abscess cavity disappeared.

Conventional surgery was performed to cut out liver abscess in the control group, followed by catheter drainage. After selecting an appropriate puncture position, the skin was disinfected and draped. The ultrasonic probe was wrapped with a sterile probe sleeve and placed in the surgical field. Under local anesthesia with 5-10 ml of 2% lidocaine at the puncture position, an incision about 0.3-0.4 cm wide was made with a sharp blade. Then, an 8Fr Skater trocar was inserted into the abscess cavity, and the internal needle was removed. The cannula was left and fixed at a relatively low point of the abscess cavity, externally connected to a sterile drainage bag. Then, 5–10 ml of pus was drawn and sent for bacterial culture for drug susceptibility testing.

The article "Efficacy and Prognosis of Ultrasound-Guided Percutaneous Catheter Drainage in Patients with Liver Abscess Complicated with Septic Shock" was retracted in 2023. Reasons: signs of a paper mill; suspected computer-generated content; unreliable results or conclusions; lack of ethics approval or compliance.

Postoperative complications such as bleeding were observed for 30 minutes. When indwelling drainage tube, the drainage volume and the color of drainage fluid were recorded daily with the drainage tube well fixed. Postoperative body temperature and white blood cell count were closely observed. The US was performed 3 days and 1 week after the operation to detect the presence of complications and abscess condition. Bacterial culture was performed on the aspirated pus, and sensitive antibiotics therapy was administered to the patients with positive bacterial culture and broad-spectrum antibiotics to negative patients based on clinical experience. The patients' blood glucose levels were strictly controlled, hypoproteinemia and water and electrolyte imbalance were corrected, and care was taken to maintain acid-base balance and assure vitamin and nutritional support. The time to return to normal body temperature, time to return to normal peripheral white blood cell count, postoperative extubation time, and postoperative hospital stay were recorded in both groups.

### 2.3. Detection of Biochemical Indicators

In both groups, blood samples were collected on an empty stomach in the morning on postoperative days 0, 2, 4, and 6. After standing at room temperature for 1.5 h, the supernatant was collected after centrifugation at 3500 rpm for 10 min. The serum levels of liver function parameters alanine aminotransferase (ALT), aspartate aminotransferase (AST), total bilirubin (TBIL), direct bilirubin (DBIL), and alkaline phosphatase (ALP) were measured using an automatic biochemical analyzer (Mindray, China).

### 2.4. ELISA

The serum levels of inflammatory cytokines interleukin 6 (IL-6), IL-8, and tumor necrosis factor *α* (TNF-*α*) were measured on postoperative days 0, 2, 4, and 6 in both groups using ELISA kits (United, China).

### 2.5. Incidence of Complications/Adverse Reactions

Complications/adverse reactions, such as infection, abdominal bleeding, abdominal abscess and severe pain, were recorded in both groups.

### 2.6. Follow-Up

The two groups were followed up for 12 months after surgery, and the survival of the patients was recorded to calculate the survival rate.

### 2.7. Statistical Methods

All data were statistically analyzed using the SPSS 24.0 software. Measurement data were expressed as mean ± standard deviation (mean ± SD), and two independent sample *t*-test was used for comparison between the two groups; enumeration data were expressed as frequency (*n*) and rate (%), and the chi-square test was used for analysis. *P* < 0.05 indicated significant difference.

The article "Efficacy and Prognosis of Ultrasound-Guided Percutaneous Catheter Drainage in Patients with Liver Abscess Complicated with Septic Shock" was retracted in 2023. Reasons: signs of a paper mill; suspected computer-generated content; unreliable results or conclusions; lack of ethics approval or compliance.

## 3. Results

### 3.1. General Information of Patients

As demonstrated in Table 1, the observation group consisted of 44 males and 26 females, with a mean age of 55.34 ± 7.78 years and an average diameter of lesions of 8.05 ± 1.17 cm. The lesions were detected in a single lobe in 48 patients and in both left and right lobes in 22 patients. Comparatively, the control group consisted of 30 males and 20 females, with an average age of 54.72 ± 8.83 years, and their average diameter of lesions was 8.16 ± 0.82 cm. Of these lesions, 36 were single, and 14 were multiple. There was no difference in gender composition ratio, age, lesion size, and location between the two groups. The difference in white blood cells, neutrophils, systolic blood pressure, and other biochemical parameters between both groups did not reach significance, indicating that the groups were comparable (Table 1).

### 3.2. Ultrasound-Guided Percutaneous Catheter Drainage Can Significantly Reduce the Extent of Liver Abscess

CT scan and color Doppler ultrasonography were performed before the operation. The results showed a quasi-circular low-density shadow in the right lobe of the liver with a clear boundary and fluid density content inside and surrounding edema. Its upper part manifested gas and an air-fluid level (Figures 1(a)–1(c)). After US-PCD, US and CT images showed that the drainage tube was in place, and the extent of the liver abscess was significantly reduced (Figures 1(d)–1(f)).

### 3.3. Ultrasound-Guided Percutaneous Catheter Drainage Can Significantly Improve Liver Function and Reduce the Level of Inflammatory Factors in Patients

We investigated the levels of liver function parameters ALT, AST, TBIL, DBIL, and ALP and inflammatory cytokines IL-6, IL-8, and TNF-*α* in both groups on postoperative days 0, 2, 4, and 6. The results showed that compared with day 0 after the operation, the serum levels of these liver function parameters in the observation group gradually decreased over time and returned to the normal range, and the recovery trend in the observation group was significantly better than in the control group (Figures 2(a)–2(h)). The results showed that US-PCD had a good therapeutic effect in patients with liver abscess.

### 3.4. Ultrasound-Guided Percutaneous Catheter Drainage Can Reduce the Recovery Time of Patients

Comparisons of postoperative recovery time between the two groups showed that the time to return to normal body temperature, time to return to normal peripheral white blood cell count, postoperative extubation time, and postoperative hospital stay in the observation group were significantly lower than the control group (Table 2). It also showed that the patients recovered quickly after US-PCD.

The article "Efficacy and Prognosis of Ultrasound-Guided Percutaneous Catheter Drainage in Patients with Liver Abscess Complicated with Septic Shock" was retracted in 2023. Reasons: signs of a paper mill; suspected computer-generated content; unreliable results or conclusions; lack of ethics approval or compliance.

### 3.5. Ultrasound-Guided Percutaneous Catheter Drainage Can Reduce the Occurrence of Adverse Reactions in Patients

The adverse reactions were further compared between the two groups. The observation group had a significantly lower incidence of adverse reactions such as infection, abdominal hemorrhage, abdominal abscess, and severe pain (Table 3). The results showed that the incidence of adverse reactions was significantly reduced after US-PCD.

### 3.6. Ultrasound-Guided Percutaneous Catheter Drainage Can Significantly Improve the Survival Rate of Patients

All patients were followed up for 12 months after the operation, and the survival rate was recorded. The results showed that US-PCD achieved a higher survival rate at 3 months, 6 months, and 12 months after operation in the observation group relative to the control group (Figure 3), indicating that US-PCD was associated with a good prognosis in the treatment of liver abscess.

## 4. Discussion

Infection of liver abscess is driven by complex causes, is common in clinical practice, and may rapidly and seriously develop. Its incidence keeps arising due to an increased incidence of diabetes and biliary tract diseases. The most common routes of infection are biliary tract infection and hematogenous infection [19]. The clinical manifestations of patients with liver abscess include fever, nausea/vomiting, chills, liver pain, elevated white blood cell count, with or without hepatomegaly, and fatigue [20, 21]. Currently, surgical treatment is advocated in clinical practice for attenuating the condition in which the puncture and drainage technique is widely used. Further, the puncture and drainage operation is simpler [22]. Some studies have suggested that US-guided puncture may reduce the incidence of complications, and its safety and effectiveness allow it to be increasingly used in clinical practice [9, 23, 24]. Studies suggest that in the case of a thick cavity wall, puncture aspiration hardly aspirates the pus completely, while puncture drainage can compensate for this defect and improve the efficacy [25]. In this study, patients with liver abscess complicated with septic shock underwent conventional surgical incision and drainage of liver abscess and US-PCD, respectively. The results suggested that US-PCD could significantly improve the clinical efficacy and reduce the stress response. Liver abscess can cause a stress response in response to inflammation resulting in decreased serum superoxide dismutase and increased serum oxidative stress mediators cortisol (COR) and malondialdehyde [26]. In the past, traditional treatment was symptomatic, the drug action time was short, and the improvement effect on stress response was poor [27]. US-PCD can accurately locate the lesion, avoid vital organs such as ribs and sternum, and reasonably control the depth of needle insertion when the position of needle insertion can be adjusted to observe the drainage status of pus [28, 29]. Drainage can achieve the purpose of bacteriostasis and sterilization when controlling the infection and facilitating the healing of the abscess cavity [30]. Therefore, compared with conservative treatment, US-PCD can further alleviate the stress response, which was consistent with the results of this present study.

The article "Efficacy and Prognosis of Ultrasound-Guided Percutaneous Catheter Drainage in Patients with Liver Abscess Complicated with Septic Shock" was retracted in 2023. Reasons: signs of a paper mill; suspected computer-generated content; unreliable results or conclusions; lack of ethics approval or compliance.

The possible disadvantages of US-PCD could be difficulties in the visualization of deeper targets, obstruction by bowel gas, and attenuation of the sound beam on larger or obese patients. However, none of these were found in this study since we mainly investigated abscesses in the liver. Compared with the control group, we found that patients in the observation group had a significantly lower incidence of adverse events such as infection, abdominal hemorrhage, abdominal abscess, and pain. Thus, this confirms the practicality of using US-PCD in clinical practice over routine surgical incisions, which were performed in the control group.

Studies have shown that the body of patients with liver abscesses is often in an inflammatory state. IL-6, IL-8, and TNF-*α* are typical inflammatory indicators, and their expressions are increased in the serum during inflammation [31, 32]. The results of this study found high serum levels of IL-6, IL-8, TNF-*α*, ALT, AST, TBIL, DBIL, and ALP before treatment in both groups, suggesting the presence of inflammation in the body. Subsequently, their levels were decreased after treatment, indicating that both regimens could alleviate inflammation. Especially lower levels were noticed in the observation group and returned to normal, indicating an anti-inflammatory effect and promoting effect on liver function of US-PCD, as this approach can reduce patients' recovery time. US-PCD can remove pus and reduce inflammatory reactions through drainage [33], which may be an important mechanism underlying its role in treating liver abscesses. Some studies also confirmed the protective role of ultrasound-guided puncture in liver function and its reliability, indicating this approach as convenient for early detection of complications and reducing the incidence of adverse events [34]. This study found that US-PCD significantly reduced patient complications and improved patient outcomes, suggesting its high safety.

The article "Efficacy and Prognosis of Ultrasound-Guided Percutaneous Catheter Drainage in Patients with Liver Abscess Complicated with Septic Shock" was retracted in 2023. Reasons: signs of a paper mill; suspected computer-generated content; unreliable results or conclusions; lack of ethics approval or compliance.

## 5. Summary

Collectively, US-PCD demonstrated a good effect in treating liver abscesses with septic shock and could significantly reduce the recovery time of patients and improve the patients' prognosis.

## Figures and Tables

**Figure 1:** Imaging of patients with liver abscess treated with ultrasound-guided puncture and drainage. (a) Preoperative CT arterial phase image of patients with liver abscess; (b) preoperative CT venous phase image of patients with liver abscess; (c) preoperative CT parenchymal phase image of patients with liver abscess; (d, e) color Doppler ultrasound image of patients with liver abscess (d) three days and (e) one week after ultrasound-guided drainage; (f) CT coronal image of patients with liver abscess after ultrasound-guided drainage.

**Figure 2:** Postoperative biochemical indicators of liver function and levels of inflammatory factors in the two groups. (a–e) Serum ALT, AST, TBIL, DBIL, and ALP levels on postoperative days 0, 2, 4, and 6 in both groups; (f–h) serum IL-6, IL-8, and TNF-*α* levels on postoperative days 0, 2, 4, and 6 in both groups. ^∗∗^*P* < 0.01*vs*. control group. ALT: alanine aminotransferase; AST: aspartate aminotransferase; TBIL: total bilirubin; DBIL: direct bilirubin; ALP: alkaline phosphatase; IL-6: interleukin 6; TNF-*α*: tumor necrosis factor *α*.

**Figure 3:** Survival of the two groups after 12 months of follow-up.

**Table 1:** Baseline characteristics of patients in the two groups.

Variable	Observation group	Control group	*t*/*χ*^2^	*P*
Gender (M/F)	44/26	30/20	0.101	0.751
Age (years)	55.34 ± 7.78	54.72 ± 8.83	0.409	0.684
Body mass index	28.10 ± 1.49	28.35 ± 2.85	0.573	0.569
Onset symptom			0.440	0.932
Fever	37	25		
Abdominal pain	12	10		
Vomiting	13	8		
Others	8	7		
Abscess diameter (cm)	8.05 ± 1.17	8.16 ± 0.82	0.615	0.540
Septic shock staging			0.876	0.645
Stage 1	31	23		
Stage 2	30	18		
Stage 3	9	9		
Infected parts (n)			0.163	0.686
Single lobe	48	36		
Both lobes	22	14		
Shock time (h)	3.20 ± 1.46	3.12 ± 1.00	0.356	0.723
White blood cell count (109/L)	18.26 ± 2.49	18.95 ± 2.24	1.570	0.119
Neutrophil percentage (%)	75.44 ± 3.77	74.39 ± 3.23	1.599	0.113
Total protein (g/L)	73.73 ± 6.65	74.00 ± 5.25	0.241	0.810
Plasma albumin (g/L)	48.30 ± 5.18	48.20 ± 3.06	0.143	0.887
Hemoglobin (g/L)	163.14 ± 8.45	160.53 ± 7.94	1.712	0.090
Blood glucose (nmol/L)	4.53 ± 0.77	4.45 ± 0.67	0.546	0.586
Total cholesterol (mmol/L)	5.11 ± 0.51	5.31 ± 0.70	1.684	0.096
Triglycerides (mmol/L)	3.23 ± 0.41	3.33 ± 0.34	1.458	0.148
High-density lipoprotein (mmol/L)	1.35 ± 0.37	1.37 ± 0.08	0.404	0.687
Low-density lipoprotein (mmol/L)	3.20 ± 0.82	3.12 ± 0.18	0.805	0.423
Systolic blood pressure (mmHg)	77.97 ± 7.64	79.04 ± 6.07	0.853	0.396
Diastolic blood pressure (mmHg)	110.26 ± 9.70	111.72 ± 9.20	0.832	0.407

The article "Efficacy and Prognosis of Ultrasound-Guided Percutaneous Catheter Drainage in Patients with Liver Abscess Complicated with Septic Shock" was retracted in 2023. Reasons: signs of a paper mill; suspected computer-generated content; unreliable results or conclusions; lack of ethics approval or compliance.

**Table 2:** Comparison of postoperative recovery time between the two groups.

Variable	Observation group	Control group	*T*	*P*
Temperature recovery time (day)	3.80 ± 0.65	5.34 ± 0.77	11.820	≤0.001
Recovery time of peripheral white blood cell count (day)	3.19 ± 0.73	5.90 ± 0.58	21.855	≤0.001
Time to extubation (days)	11.46 ± 1.59	15.34 ± 1.95	11.963	≤0.001
Postoperative hospital stay (days)	15.94 ± 1.89	20.86 ± 2.28	12.903	≤0.001

**Table 3:** Incidence of adverse reactions in the two groups.

Variables	Observation group	Control group	*χ* ^2^	*P*
Infection	2 (2.86)	10 (20.00)	9.521	0.002
Abdominal hemorrhage	3 (4.29)	15 (30.00)	12.455	≤0.001
Abdominal abscess	5 (7.14)	11 (22.00)	5.571	0.018
Intense pain	1 (1.43)	9 (18.00)	8.380	0.004

## Data Availability

The data used to support the findings of this study are available from the corresponding author upon request.
